# Prior Distribution Estimation of Monitored Information in the Intensive Care Unit with the Hidden Markov Model and Decision Tree Methods

**DOI:** 10.1155/2022/7892408

**Published:** 2022-03-24

**Authors:** Xin Zhao, Xiaokai Nie, Guofei Pang, Siyuan Qiu, Kehan Shi, Changqing Wang, Bingqi Zhao, Yidan Huo

**Affiliations:** ^1^School of Mathematics, Southeast University, Nanjing 211189, China; ^2^School of Automation, Southeast University, Nanjing 210096, China; ^3^Key Laboratory of Measurement and Control of Complex Systems of Engineering, Ministry of Education, Southeast University, Nanjing 210096, China; ^4^Shenzhen Research Institute, Southeast University, Shenzhen 518057, China

## Abstract

In the intensive care unit, the monitored variables collected from sensors may have different behaviors among patients with different clinical basic information. Giving prior information of the monitored variables based on their specific basic information as soon as the patient is admitted will support the clinicians with better decisions during the surgery. Instead of black box models, the explainable hidden Markov model is proposed, which can estimate the possible distribution parameters of the monitored variables under different clinical basic information. A Student's *t*-test or correlation test is conducted further to test whether the parameters have a significant relationship with the basic variables. The specific relationship is explored by using a conditional inference tree, which is an explainable model giving deciding rules. Instead of point estimation, interval forecast is chosen as the performance metrics including coverage rate and relative interval width, which provide more reliable results. By applying the methods to an intensive care unit data set with more than 20 thousand patients, the model has good performance with an area under the ROC Curve value of 0.75, which means the hidden states can generally be correctly labelled. The significant test shows that only a few combinations of the basic and monitored variables are not significant under the 0.01 significant level. The tree model based on different quantile intervals provides different coverage and width combination choices. A coverage rate around 0.8 is suggested, which has a relative interval width of 0.77.

## 1. Introduction

In the intensive care unit (ICU), patients suffer from complications like sepsis and circulatory failure during surgery. Such complications will incur serious conditions out of medical control [1, 2]. Without fast and accurate disease diagnosis, patients face a high death rate due to lack of proper treatment. To improve the diagnosis efficiency, a prior information extraction method was developed in this research. As soon as the patients are admitted into the ICU, their basic clinical data can be checked from the medical information system. By giving the prior probability calculated from the basic clinical data, it can improve the posterior probability either diagnosed by the surgeons or by models like Bayesian.

The model developed during the training process in this research utilizes the basic clinical data before the surgery and the monitored data during the surgery. The data include two parts (1) the basic clinical data *B*_*n*,._ for patient *n* including variables such as sex, age, weight, and height.

(1) $$\begin{array}{c} B_{n,\cdot }=\left[B_{n,1},B_{n,2},\ldots ,B_{n,k},\ldots \right], \end{array}$$

where *n*=1,2,…, *N* and *k*=1,2,…, *K*. (2) The monitored data during the surgery for patient *n*, including variables such as heart rate and cardiac output.

(2) $$\begin{array}{c} A_{n,\cdot ,\cdot }=\left[\begin{array}{ccc} A_{n,1,1} & \cdots & A_{n,K,1}\\ A_{n,1,2} & \cdots & A_{n,K,2}\\ \vdots & \ddots & \vdots \\ A_{n,1,T_{n}} & \cdots & A_{n,K,T_{n}} \end{array}\right], \end{array}$$

where *A*_*n*_ refers to the matrix for the *n*^th^ individual containing all variables at all times. As the time length for patients differ, *T*_*n*_ is used to measure the time length for patient *n*. Without any extra information, the data for patient *n* are {*B*_*n*,·_, *A*_*n*,·,·_}.

For diseases such as circulatory failure and sepsis during surgery, there are typical methods to diagnose their onset. For example, systemic inflammatory response syndrome (SIRS) and sequential organ failure asses (SOFA) are designed for sepsis detection. These are simple decision rules by including criteria like that the temperature is higher than 38 or lower than 36. These criteria are the general diagnosis standard when patients show obvious symptoms. In the early diagnosis of neonatal sepsis, the semiquantitative PCT test kit helps to exclude negative results [3]. Cheadle et al. [4] have surveyed a number of host defense parameters that pertain to an adequate immune response and developed an outcome predictive score, which can identify patients within hours of hospitalization who are at risk of subsequently developing overt clinical infection and sepsis. For observations *A*_*n*,·,*t*_ at time *t*, a response can be given according to the diagnosis standard as *y*_*n*,*t*_. Until now, the data for patient *n* are {*B*_*n*,·_, *A*_*n*,·,·_, *y*_*n*,·_}.

The current research for disease analysis by using the abovementioned data can be divided into three aspects, which are as follows:

1. The relationship analysis of basic clinical data *B* and response variables such as survival rate. The models can be traditional biostatistics tests and machine learning methods [5]. For example, Chicco and Jurman [6] predict the survival rate of patients with sepsis from age, sex, and septic episode number alone.
2. From the static aspect, the data *A* is regarded as a static multivariate time series, which assumes the data follow the same distribution without changing with time, thus a stationary process. Methods such as neural networks or ensemble learning technics such as the random forest or AdaBoost are used in the modeling process [7].
3. From the dynamic aspect, the time series are regarded as dynamic multivariate variables, thus a nonstationary process [8]. Dynamic models are designed by giving model updating or retraining criteria. For example, Zhao et al. [9] use wavelet transform and decision tree-based methods to do interval forecasting for monitored data *A*. The input variables involved include *A* and sometimes *B*. For example, Esteban et al. [10] predict clinical events by combining static and dynamic information using recurrent neural networks. The data *B* is involved as an input layer in the neural network, resulting in an improvement in the performance. Bernhardt [11] proposes a two-part regression model composed of logistic regression and a truncated accelerated failure time model, which helps to use all of the available survival information. Instead of involving the data *B* in the existing model, Lin et al. [12] built a separate model to train *B* and combined it with the convolutional long short-term memory neural networks trained for *A*. In addition to the data *A* and *B*, pharmacy data are also used in the modeling process, as demonstrated by Hyland et al. [13].

Current research mainly concentrate on one specific disease with two states being safe or onset. But the reality is that multiple states may occur during the surgery process. Prediction of one specific state may reduce the data information utility and ignoring other states may bring more uncertainty to the health condition of the patients. In addition, the criteria of disease onset detection like SIRS may not cover all possible hidden conditions. The states can be regarded as hidden states that are not seen or cannot be measured directly while the monitored variables like *A* or basic information *B* are not hidden. One of the main hidden states model is the hidden Markov model. Christopher et al. give the initial probability distribution calculation method of the multi-Markov model for such data. Their following research can be seen from Christopher, Ieva et al. [14]. In this case, hidden state models are proposed in this research to label the state for each observation of each patient.

The distribution of data *A* is rarely studied among the researches, as most of the methods are nonparametric methods which have no parameter assumptions like some of the machine learning methods. But if the distributions can be estimated, the correlation of the basic clinical data *B* and the distributions of different state labels can be established. In that case, by giving the prior information of *B*, the clinicians can have the estimated posterior distribution of *A* of different disease states. For example, if females have an average higher heart rate than males, a heart rate value normal for females may be alerted for males. If the heart rate is not distinguished by sex, male patients may be delayed in medical treatment. So, in this research, the distributions of monitored data *A* are studied under different states' labels. The correlation between distribution parameters and basic clinical data is tested to distinguish their differences among different basic information.

The innovative aspects in this paper include the following: (1) the multivariable hidden Markov model is selected to discover the hidden states that may not be measured by the general standard rules. (2) The variables' distribution of *A* labelled with different states is estimated by the hidden Markov model under the Gaussian assumption. (3) The variables' distributions are compared under different prior basic clinic conditions to give a posterior information for clinical decision.

We introduce our basic model in Section 2, and apply it to the real data in Section 3. Some concluding comments appear in Section 4. All calculations were carried out using R Core Team [15]; “depmmixS4” [16] was used for the hidden Markov model and “ctree” by Hothorn et al. [17] for the Ctree.

## 2. Methods

The hidden Markov model (HMM) origins from the research [18] for discrete observations and is further developed for time series; detailed study was carried out in [19]. The HMM has observations which are observable, such as the monitored variable heart rate which can be collected by sensors. The observations are generated by the corresponding states which are not observable, like the status of the patient as sick or healthy, as circulatory failure or normal. The HMM has three typical questions: likelihood, decoding, and learning. What is used in this research are decoding and learning, which are finding the most likely hidden status and learning the parameters of the model.

If the distribution of the observations are assumed to be Gaussian distribution, for patient *n* and monitored variable *k* at status *s*, by giving the parameters of initial distribution as *π*_*s*_, Gaussian distribution as *μ*_*n*,·,*s*_, Σ_*n*,·,*s*_, the conditional joint distribution is

(3) $$\begin{array}{c} f\left(A_{n,\cdot ,\cdot },y_{n,\cdot }|\pi_{s},\mu_{n,k,s},\sigma_{n,k,s}\right)=\prod_{t=1}^{T_{n}}\prod_{k=1}^{K}\pi_{s}^{I\left(y_{n,t}=s\right)}N{\left(A_{n,k,t}|\mu_{n,\cdot ,s},\Sigma_{n,\cdot ,s}\right)}^{I\left(y_{n,t}=s\right)}, \end{array}$$

where *I*(*y*_*n*,*t*_=*s*) is the indicator variable showing whether the status of patient *n* at time *t* is *s* or not. If the variables are further assumed to be independent mutually, then the distribution is

(4) $$\begin{array}{c} f\left(A_{n,\cdot ,\cdot },y_{n,\cdot }|\pi_{s},\mu_{n,k,s},\sigma_{n,k,s}\right)=\prod_{t=1}^{T_{n}}\prod_{k=1}^{K}\pi_{s}^{I\left(y_{n,t}=s\right)}{\left\{\prod_{k=1}^{K}N\left(A_{n,k,t}|\mu_{n,k,s},\sigma_{n,k,s}\right)\right\}}^{I\left(y_{n,t}=s\right)}. \end{array}$$

By using the Baum–Welch algorithm (expectation maximization algorithm) and assuming the initial distribution is equally distributed, the Gaussian distribution parameters can be estimated for patient *n*, variable *k*, and state *s* as follows:

(5) $$\begin{array}{c} \left\{{\hat{\mu }}_{n,k,s},{\hat{\sigma }}_{n,k,s}\right\}. \end{array}$$

By applying the forward-backward algorithm, the best hidden states ${\hat{y}}_{n,t}$ and its corresponding probability *p*(*y*_*n*,*t*_=*s*) can be estimated.

Since the hidden states are discrete, the metric AUC (area under the ROC curve) is chosen to measure the similarity between the real and estimated hidden states. A ROC curve (receiver operating characteristic curve) is a graph showing the performance of a classification model at all classification thresholds. AUC provides an aggregate measure of performance across all possible classification thresholds, which ranges in value from 0 to 1. A model whose predictions are 100 % wrong has an AUC of 0.0; one whose predictions are 100 % correct has an AUC of 1.0, while random guessing has an AUC of 0.5.

If the AUC results are acceptable, the estimated parameters $\left\{{\hat{\mu }}_{n,k,s},{\hat{\sigma }}_{n,k,s}\right\}$ can be reliable. After that, the parameters are compared under different basic clinical data *B*. For example, the data ${\hat{\mu }}_{\cdot ,k,s}$ of variable *k* and state *s* are compared under different sex to test whether it has significant difference between female and male patients. The comparing methods include Student's *t*-test for discrete variables such as sex and the correlation test for continuous variables such as age, weight, and height. If the test shows significant results, the model decision tree is further conducted to find how the basic clinical variable influences the monitored variables' distribution, namely, the estimated parameters.

The model decision tree is a model of tree-like decision rules, which splits the sample space into subspaces by choosing the best split each time. Specifically, the model used in this research is a conditional inference tree (Ctree [17]). Ctree estimates a regression relationship by binary recursive partitioning in a conditional inference framework. The predictor variable, like the clinical basic variables, with the lowest p value is selected for splitting the response variable, for example, ${\hat{\mu }}_{\cdot ,k,s}$ of variable *k* and state *s*. The p value belongs to a split criterion which can be Spearman's correlation test, the Wilcoxon–Mann–Whitney test, the Kruskal–Wallis test, permutation tests, and so on. The stoping criteria are not constrained to the p value, but also include the max tree depth allowance. For example, a max tree depth of 5 means the tree can be no bigger than 5 in depth. Other stopping criteria may also be applied. A regression tree is formed by iteratively splitting nodes so as to maximize the decreased p value at each step.

For each observation, it will be split into one single terminal node. The observations in the same terminal node can be regarded as a set. By ranging the *Y* values in that set, the quantile values can be selected as the forecast interval. For example, an 80 % interval has an upper value of 0.9 quantiles and a lower value of 0.1 quantiles. The width of the quantile interval is further standard adjusted to remove the influence of the different variable units by dividing their 0.9 quantile difference of the variable.

(6) $$\begin{array}{c} \text{Relative interval width}=\frac{\text{original interval width}}{\text{0.}95\text{ quantile}-\text{0.}05\text{ quantile}}. \end{array}$$

The coverage of the interval is as follows:

(7) $$\begin{array}{c} \text{coverage rate}=\frac{\text{number of observations in the interval}}{\text{total number of observations}}. \end{array}$$

A wider interval has a high coverage when a new observation comes into the same terminal node, but at the cost of a higher width. An interval with good coverage and suitable width is suggested.

## 3. Real Data Analysis and Results

In the real data analysis, the circulatory failure data from Hyland et al. [13] are used. After deleting patients who have missing values, the data contains 22290 patients. The data include monitored variables A such as heart rate, systolic blood pressure (BP), diastolic BP, mean arterial pressure (MAP), and basic clinical data B such as sex, age, weight, height, and body mass index (BMI). Sepsis is a systemic inflammatory response syndrome caused by the invasion of pathogenic microorganisms such as bacteria into the body. Associated dysregulation of the inflammatory response has been thought to be directly associated with cardiomyocyte dysfunction. And heart rate reflects the frequency with which cardiomyocytes move. Systolic BP, diastolic BP, and MAP are related to blood volume, elasticity and tension of blood vessel walls, and cardiac output. They can all reflect well the ability of cardiomyocytes and can serve as an indicator of sepsis. For the state variable *y*, it is labelled generally according to the rule from [13]: *y*_*n*,*t*_ is labelled as circulatory failure if MAP is ≤65 mmHg or (not exclusive) vasoactive/inotropic drugs are present and lactate is bigger than 2 mmol l^−1^. Under the other circumstances, *y*_*n*,*t*_ is labelled as safe.

For the data *A*_*n*,·,·_ of patient *n*, we train them with the model HMM under the Gaussian distribution assumption. The estimated states and the estimated parameters for the variable heart rate of one patient example are shown in Figure 1.

(8) $$\begin{array}{c} {\hat{y}}_{n,t}=f\left(A_{n,\cdot ,\cdot }\right). \end{array}$$

One thing that needs to be noticed is that the hidden state of not being safe is not constrained to circulatory failure but may also include others. The reason *y*_*n*,*t*_ is labelled as circulatory failure is because circulatory failure is the main disease during the process. If it can be correctly labelled, the HMM results can be reliable. After the HMM processing, the AUC value is calculated for patients who have multiple states in *y*_*n*,_. The patients with only circulatory failure or safe state, namely, *y*_*n*,_ with only one label, are not involved in the AUC measurement. After that, the number of patients is 10406. The histogram of the results is shown in Figure 2.

The result shows that, the HMM model can efficiently recognize the patterns of the data, thus most of the states are labelled with the right tag. Since the AUC results are acceptable, the estimated parameters $\left\{{\hat{\mu }}_{n,k,s},{\hat{\sigma }}_{n,k,s}\right\}$ can be reliable. After that, the *t*-test or correlation test is conducted to test whether the estimated ${\hat{\mu }}_{n,\cdot ,s}$, ${\hat{\Sigma }}_{n,\cdot ,s}$ have significant difference among different basic clinical settings. The results are shown in Table 1.

The results show that most of the parameters have a significant correlation with the clinical basic variables. By giving the clinical basic information, the parameters can have their values estimated, which can be regarded as the prior values for the monitored variables. Instead of point estimation, interval estimation is suggested to give more reliable support for clinicians. The model Ctree is applied, with the threshold chosen as 0.1 and the tree max depth as 5, which balances the performance and complexity of the model. For example, when the forecast interval is set as 84 %, the coverage rate and relative width across the 32 monitored variables are shown in Figure 3.

Since the correlation significant results differ across the monitored variables, the coverage rate and relative interval width have different performances. But the results are relatively acceptable as they are generally around 0.84, the preset forecast interval.

When the forecast interval changes, the averaged coverage rate and averaged relative interval width can be estimated. The results are shown in Figure 4. It can be shown that when the interval width increases, the coverage rate also increases, but at a decreasing speed. An increase of 0.1 may cost the width of 0.5 when coverage has reached 0.8. A result of around 0.8 is proposed, which has relatively high coverage but not that wider width. It should be noted that this study involves one disease, sepsis, but includes different stages of sepsis and has a large sample size to support the data, so the model is stable and can be generalized.

## 4. Conclusion

In order to calculate the prior distribution parameters of the monitored variables of different hidden states, this research gives a method by using the explainable HMM and Ctree models. The HMM finds the most possible hidden states, and the estimated states are compared with the true circulatory failure states, which results in an AUC of 0.75 in the real data analysis. Thus, the distribution parameters of the monitored variables learned by the HMM can be reliable. The *t*-test or correlation test is applied to test the significant relationship between the basic clinical variable and the distribution parameters of the monitored variables. Results show that most relationships are significant, which means the distribution of the monitored variables truly has some kind of dependence on the clinical basic information. To further explore the specific relationship, the model Ctree is conducted. Instead of point estimation, interval forecast is applied, along with the coverage rate and relative interval width as the performance metrics. Results show that, with a wider width, the coverage increases. But the increase decays when the coverage reaches a high level. A good coverage of 0.8 with a suitable width is suggested.

In further research, in terms of the method, the parameters of the monitored variables can be assumed to follow different distributions without being constrained to follow a Gaussian distribution. This can help extend the method for more general conditions. In terms of the variable relationship exploration part, the relationship test can be applied to a mixture of variables instead of one at a time. This helps explore more potential relationships among different variables. In the interval forecast method, point estimation can be conducted by including other input variables so as to get a good performance. In terms of sepsis, as it is a threat to the public health with high morbidity and mortality, further research can be extended from diagnosis assistance to also include prevention and treatment support. More machine learning methods can be developed to solve the potential problems incurred by the rapid development of medical technology.

The results of the research can not only be used for clinician support but also provide prior distribution for the models of state prediction during the monitoring process. This can improve the prediction accuracy at the beginning of the prediction process. If further pharmacy information is added, the research can also be used for exploring the influence of clinical basic information in the usage of drugs. Suitable and timely drug dosage provides the possibility of precision medicine. By combining machine learning technologies with medical demand, medical problems can be solved more automatically by modern algorithms, and less human resources are required. The method developed in this research can be also applied in other areas such as financial and economical areas, environmental regulation, and so on.

## Figures and Tables

**Figure 1:** The hidden Markov model (HMM) result for one patient with multiple states. In the first figure, the HMM estimated red (below the black line) points are generally consistent with the black points (above the red line). Its corresponding AUC value is 0.8962. In the second figure, the right red Gaussian curve has the parameters *μ*=95.675 and *σ*=10.027, and the left black curve has the parameters *μ*=87.123 and *σ*=8.918. The observations of state circulatory failure have a relatively lower *μ*.

**Figure 2:** The area under the ROC curve (AUC) results for patients with multiple states. The AUC value of 0.5 means the model has a performance of random guessing. A value higher than that means the model has better performance.

**Figure 3:** The coverage rate and relative interval width of the 32 monitored variables under the 84% forecast interval. The averaged relative interval width is 0.77, and the averaged coverage rate is 0.81.

**Figure 4:** The averaged coverage rate and relative interval width of the 32 monitored variables under different forecast intervals.

**Table 1:** The *p* value of the *t*-test or correlation test.

Variable	Heart rate				Systolic BP (invasive)				Diastolic BP (invasive)				MAP			
Parameter	*μ*		*σ*		*μ*		*σ*		*μ*		*σ*		*μ*		*σ*	
State	1	2	1	2	1	2	1	2	1	2	1	2	1	2	1	2
Sex	0.028	0.026	0.000	0.000	0.027	0.047	0.132	0.604	0.152	0.463	0.446	0.051	0.000	0.000	0.024	0.001
Age	0.000	0.000	0.000	0.000	0.309	0.365	0.000	0.000	0.000	0.000	0.001	0.000	0.000	0.000	0.000	0.000
Weight	0.113	0.163	0.000	0.000	0.029	0.025	0.000	0.001	0.000	0.001	0.000	0.008	0.023	0.014	0.022	0.325
Height	0.000	0.000	0.002	0.000	0.010	0.002	0.481	0.362	0.000	0.000	0.052	0.483	0.372	0.183	0.111	0.000
BMI	0.000	0.000	0.000	0.000	0.487	0.788	0.000	0.000	0.097	0.006	0.000	0.006	0.000	0.000	0.000	0.014
Variable	Cardiac output				SpO2				INR				Serum glucose			
Parameter	*μ*		*σ*		*μ*		*σ*		*μ*		*σ*		*μ*		*σ*	
State	1	2	1	2	1	2	1	2	1	2	1	2	1	2	1	2
Sex	0.000	0.000	0.000	0.000	0.001	0.000	0.610	0.895	0.667	0.434	0.531	0.130	0.014	0.000	0.000	0.000
Age	0.000	0.000	0.000	0.000	0.000	0.000	0.000	0.000	0.000	0.000	0.000	0.000	0.000	0.000	0.000	0.000
Weight	0.000	0.000	0.000	0.000	0.000	0.000	0.462	0.814	0.425	0.754	0.168	0.004	0.000	0.000	0.004	0.037
Height	0.000	0.000	0.000	0.000	0.019	0.001	0.863	0.999	0.218	0.097	0.195	0.007	0.000	0.014	0.000	0.000
BMI	0.000	0.000	0.000	0.000	0.000	0.000	0.312	0.783	0.585	0.552	0.280	0.066	0.000	0.000	0.000	0.000

BP: blood pressure MAP: mean arterial pressure BMI: body mass index INR: international normalized ratio.

## Data Availability

The source codes in the methods are available from the corresponding author upon request. The real data in the application can be requested from Hyland et al. [13] [20, 21].
